The article "Prognostic Value of Creatine Phosphate and Inflammatory Markers for Mitral Valve Replacement: A Systematic Review and Meta-Analysis" was retracted in 2023. Reasons: signs of a paper mill; suspected computer-generated content; unreliable results or conclusions; concerns about the data.

# Prognostic Value of Creatine Phosphate and Inflammatory Markers for Mitral Valve Replacement: A Systematic Review and Meta-Analysis

**DOI:** 10.1155/2022/1132452

**Published:** 2022-03-11

**Authors:** Yanhui Zhu, Chengwei Zou, Jun Zhang, Lei Chen, Yanting Jia

**Affiliations:** ^1^Department of Cardiac Surgery, Shandong Provincial Hospital, Cheeloo College of Medicine, Shandong University, Jinan, 250021 Shandong, China; ^2^Department of Cardiac Surgery, Shandong Provincial Hospital Affiliated to Shandong First Medical University, Jinan, 250021 Shandong, China

## Abstract

**Purpose:**

The prognosis of mitral valve replacement is an important clinical issue and may produce unexpected mortality rates if not properly addressed. The postoperative examination results have important prognostic implications. This study was designed to determine the prognostic value of phosphocreatine and inflammatory markers after mitral valve replacement.

**Method:**

Comparison and analysis of the data obtained using SPSS software. The computer retrieved PubMed, Science Citation Index (SCI), Embase, VIP, CNKI, CBM, and Wanfang database and manually retrieved randomized controlled trials (RCTs) published at home and abroad on the central muscle protection role of creatine phosphate in heart valve replacement, and the search period was established until February 2018. Two random literature reviewers independently screened the literature and extracted data, using Review Manager (RevMan) (Computer program), version 5.3 (The Nordic Cochrane Centre, The Cochrane Collaboration, Copenhagen, 2014). RevMan software version 5.0 assesses the risk of bias for inclusion in studies. The software performs a meta-analysis of the obtained data.

**Results:**

Ten RCTs with a total of 464 participants were enrolled. The meta-analysis results showed that (1) elevated creatine kinase levels often predict a better prognosis after mitral valve replacement (RR = 1.36, 95% CI: 1.22 to 1.52, *P* < 0.00001), (2) the creatine kinase isoenzyme level in the venous blood of the phosphocreatine group after 24 h of aortic blocking was significantly lower than that in the control group (SMD = −2.90, 95% CI: -5.19 to -0.60, *P* = 0.01), and (3) Troponin I levels were significantly lower in the intravenous creatine group than in the control group 24 h after opening of the aortic block (SMD = −1.49, 95% CI: -2.02 to -0.97,*P* < 0.00001).

**Conclusions:**

Creatine phosphate and inflammatory factor have good predictive value for the prognosis of mitral valve replacement.

## 1. Introduction

Mitral stenosis usually progresses slowly, with an average annual decrease in mitral orifice area of 0.01 cm^2^. Because of its insidious onset and long course of disease, it is difficult to detect in time, which affects early treatment and often progresses to chronic or even severe valvular heart disease [1]. For such diseases, medical treatment can only be for atrial fibrillation and the prevention of thromboembolic comorbidities and cannot reverse the pathological changes of the valves, and the early stage of the lesion can be achieved by valvuloplasty can obtain satisfactory efficacy, but when the lesion is serious, only valve replacement can be used, and mitral valve replacement is still an effective means of treating rheumatic mitral stenosis, which can significantly alleviate clinical symptoms and improve cardiac function [2, 3]. It can also prolong the life of the patient [4, 5].

The article "Prognostic Value of Creatine Phosphate and Inflammatory Markers for Mitral Valve Replacement: A Systematic Review and Meta-Analysis" was retracted in 2023. Reasons: signs of a paper mill; suspected computer-generated content; unreliable results or conclusions; concerns about the data.

### 1.1. Statement of the Problem

Reconstruct valve function to avoid accidental death.

### 1.2. Indications and Contraindications for Mitral Valve Replacement

#### 1.2.1. Indications

These are the following indications: (1) mitral stenosis and severe calcification; (2) mitral stenosis, severe valve contracture, and severe subvalvular lesions that cannot be repaired by surgery, (3) mitral stenosis and insufficiency, which cannot be solved by surgery; and (4) simple mitral insufficiency that cannot be corrected by surgery [6].

#### 1.2.2. Contraindications

These are the following contraindications: (1) Rheumatic activity was not controlled or controlled for less than 3 months; (2) patients with heart failure complicated with myocardial ischemic damage, such as advanced patients with aortic stenosis; (3) patients whose liver, kidney function, or general condition is too poor to undergo surgery; and (4) patients with bacterial endocarditis with sepsis and multiple infections should not be operated on [7].

Selection of artificial heart valve is as follows: what kind of artificial valve should be used in valve replacement surgery that should be analyzed according to the specific situation? We should consider the patient's age, occupation, physical strength and mental state, the patient's opinions on valve selection, the patient's myocardial condition, and whether the patient can receive long-term anticoagulant therapy [8, 9].

### 1.3. Prognostic Determinants for Recovery

1. Patients with mechanical valve replacement need to take anticoagulants for life (usually warfarin), regularly go to the hospital to recheck Pt, and monitor the anticoagulant effect. The patients with biological valve replacement were gradually reduced after taking anticoagulants for 3 ~ 6 months and stopped within 1 ~ 2 weeks
2. Special problems during anticoagulation: in case of black stool, hematuria, hemoptysis, gum bleeding, syncope, hemiplegia or sudden dull pain in precordial area, go to the nearest hospital for examination and treatment immediately. Injuries should be avoided. In case of injury or surgery, the receiving doctor should be informed that anticoagulants are being taken. If pregnancy is needed, contact the hospital in advance to adjust the anticoagulation scheme
3. Antibiotics should be used in time during tooth extraction, urethral dilatation, catheterization, and enteroscopy because bacteria are easy to reproduce at the artificial valve, resulting in artificial valve endocarditis. Infectious diseases such as skin furuncle and tonsillitis should be treated in time
4. After heart valve surgery, the recovery of cardiopulmonary function generally takes 6 months to 1 year. Therefore, it is generally considered to resume work after 6 ~ 8 months of rest, and the labor intensity and workload increase gradually. Patients with cardiac function reaching grade I can gradually stop cardiac stimulants and diuretics and return to normal work, but strong physical labor should be avoided. Patients whose cardiac function cannot reach grade I should continue to take cardiac stimulants and diuretics and engage in less intensive work according to their own conditions

The article "Prognostic Value of Creatine Phosphate and Inflammatory Markers for Mitral Valve Replacement: A Systematic Review and Meta-Analysis" was retracted in 2023. Reasons: signs of a paper mill; suspected computer-generated content; unreliable results or conclusions; concerns about the data.

## 2. Methods

### 2.1. Inclusion Criteria Study Type

Randomized controlled trial (RCT) is as follows: adult patients undergoing heart valve replacement for the first time in the context of external circulation, ethnicity, nationality, gender, and course of illness are not limited. Outcome index is as follows: (1) the self-synchronization rate of visceral electrical activity in the operation center was better, (2) aortic blockade opens 24 h after the phosphate creatine group of venous blood creatine kinase isoenzyme (creatine kinase isoenzyme, CK-MB) level, and (3) aortic blockade opens 24 h after the creatine phosphate group of venous blood myocardial troponin I (cardiac troponin I, cTnI) level [10–12].

### 2.2. Exclusion Criteria

These are the following factors of the exclusion criteria: (1) interventions do not meet, (2) the test object does not match, (3) studies that are repeatedly published or have similar information, (4) overview and summary, and (5) documents for which data cannot be extracted.

### 2.3. Literature Retrieval Strategy

English database retrieval strategy is as follows: subject words and free words are used for retrieval. The search words are as follows: “rheumatic heart disease,” “creatine phosphate,” “mitral valve pair,” “valvuloplasty,” and “valve replacement”. Chinese key words are as follows: “rheumatic heart disease,” “mitral valvuloplasty,” “creatine phosphate,” “mitral valve replacement”, and the references included in the literature and the compilation of academic conference papers, etc.

The article "Prognostic Value of Creatine Phosphate and Inflammatory Markers for Mitral Valve Replacement: A Systematic Review and Meta-Analysis" was retracted in 2023. Reasons: signs of a paper mill; suspected computer-generated content; unreliable results or conclusions; concerns about the data.

### 2.4. Statistical Methods

The literature quality was evaluated according to the bias risk table recommended by Cochrane Handbook 5. The included studies were retrospective clinical studies and nonrandomized blind method; so, there is the possibility of selective bias. RevMan 5.3 software and Stata 12.0 software provided by the Cochrane Collaboration Network are used for statistical analysis. Odds ratio (or) or relative risk (RR) and its 95% confidence interval (95% CI) are used as effect analysis statistics for classified data, and mean difference (MD) or standardized mean difference (SMD) and its 95% CI are used as effect analysis statistics for quantitative data. *Z*-test was used to infer the combined effect. The statistical inference of heterogeneity between included research results was *Q*-test and *I*^2^. Funnel plot was used to detect publication bias, and Begg rank correlation and egger linear regression were used to quantitatively detect publication bias. The difference was statistically significant with *P* < 0.05.

### 2.5. Postsurgical Evaluation for Prognostic Values

Preoperative routine examination is as follows: all patients underwent preoperative routine examination of cardiac color Doppler ultrasound (using GE ultrasoundvivid-7 cardiac color Doppler ultrasound, taking the apical 4-chamber section according to the method of American Society of echocardiography, and calculating the LVEF at rest by using the improved Simpson plane method), ECG, and chest film. Sample collection is as follows: all subjects fasted for 12 hours and fasting venous blood in lying position in the morning. For the detection of creatine phosphate, it is necessary to quickly inject it into the 4°C precooled enzyme inhibitor anticoagulant tube (containing 0.3 mol/l disodium EDTA) *μ*L and 0 34 mol/L (8-hydroxyquinoline 50 *μ*L and 0 32 mol/L of dimercaptopropanol 25 *μ*L). No anticoagulation is required for the detection of CRP and IL-6. Centrifuge at 3000 rpm (the high-speed centrifuge adopts Beckman company of Germany) for 5 min. The separated serum samples are stored at -30°C for batch detection. Creatine phosphate and IL-6 are analyzed by radioimmunoassay (the reagent is provided by Suzhou Aijie Biotechnology Co., Ltd.); CRP was measured by rate scattering turbidimetry (kit provided by German Deling company). Olympus AU5400 automatic biochemical analyzer is operated by professional inspection technicians according to reagent operation instructions. As noted above, these inflammatory blockages may be important for studying the recovery of the heart after changing behaviors. Infection is often essential for increasing the chances and improving over time for recovery and early detection of movement. With these unique characteristics and inflammatory features, it is easy to predict the complexities mentioned in our initiatives.

The article "Prognostic Value of Creatine Phosphate and Inflammatory Markers for Mitral Valve Replacement: A Systematic Review and Meta-Analysis" was retracted in 2023. Reasons: signs of a paper mill; suspected computer-generated content; unreliable results or conclusions; concerns about the data.

## 3. Results

In literature search results after resisting 367 articles obtained from the initial screening, 10 RCT words were finally included. A total of 464 patients were included, including 233 cases in the creatine phosphate group and 231 cases in the control group. The literature screening process and results are shown in Tables 1 and 2. The basic features of the included studies are shown in Figure 1.

### 3.1. Meta-Analysis Results

Literature of 9 RCTs was included (Figure 2). There was no statistical heterogeneity between the groups (cadaver = 29%), fixed-effect model was used, and the results showed that the intraoperative cardiac autorepulsion rate in the creatine phosphate group was significantly higher than that in the control group (1.36, 95% CI: 1.22-1.52, *P* < 0.00001), see Figure 3.The levels of serum IL-6 and IL-10 after operation were significantly lower than those before operation, and the level of IL-10 was higher than that before operation (*P* < 0.05), The score of postoperative quality of life in this group was significantly higher than that before operation (*P* < 0.05). With the increase of age, the function of various organs of the human body appears progressively degraded. Therefore, sensitivity analysis of the studies with the largest mean age excluded from the analysis showed that the difference in pooled effect values of the largest average age of patients was still statistically significant ((RR) = 1.40, 95% CI: 1.25-1.58, *P* < 0.00001).  Table 3 shows the statistical data of prognostic factors.

Aortic blockade after 24 h of venous blood CK-MB level was included in 3 RCTs. The results between the groups were statistically heterogeneous (*I*^2^ = 93%), using a random effects model, and the results showed that venous blood levels in the creatine phosphate group after opening 24 h after the opening of the aortic block were lower than in the control group (SMD = −2 90, 95% CI: -5.19--0.60, *P* = 0.01), see Figure 4.

## 4. Discussion

Mitral stenosis belongs to critical valvular disease. There are many cases in China and few reports abroad. With the improvement of people's living standard, improvement of nutritional status, progress of medical and health conditions, and the wide application of antibiotics, the incidence rate of rheumatic fever and rheumatic heart disease is decreasing, but the etiology of adult heart valve disease is still mainly rheumatic heart disease. In rheumatic heart disease, mitral stenosis is the most common [13]. Small left ventricle is considered to be an adaptive change caused by the reduction of left ventricular volume load (preload) after chronic mitral stenosis. The left ventricle is chronically insufficient for a long time, the work done is correspondingly reduced, and the cardiac output is reduced, resulting in partial myocardial fibrosis and different degrees of disuse atrophy, resulting in the occurrence of small left ventricle. Echocardiography showed that LVEDVI and LVEDD decreased significantly. Some scholars also believe that long-term rheumatic mitral valve diseases, such as mitral lobe fibrosis, hypertrophy, stiffness, contracture, tendon and papillary muscle fusion and shortening, resulting in changes in left ventricular geometry, and reduced compliance, are the main reasons for the reduction of left ventricular volume and end diastolic diameter [14]. At present, valve replacement is the main treatment for patients with mitral stenosis complicated with small left ventricle, but the perioperative mortality and postoperative complications are high. Therefore, the recovery of cardiac morphology and function after mitral valve replacement is worthy of attention [15].

The article "Prognostic Value of Creatine Phosphate and Inflammatory Markers for Mitral Valve Replacement: A Systematic Review and Meta-Analysis" was retracted in 2023. Reasons: signs of a paper mill; suspected computer-generated content; unreliable results or conclusions; concerns about the data.

Compared with before operation, left ventricular fractional shortening (LVFS) had no significant change within 2 weeks after operation and increased significantly by 6.21% after half a year, indicating that the left ventricular systolic function of these patients recovered well after operation. LVEF decreased by 3.05% within 2 weeks and increased by 7.69% half a year after operation, but the difference was not statistically significant [16]. The reasons for the insignificant changes of cardiac function indexes in the near future after operation are as follows: (1) the baseline values of LVEF and LVFS in patients with mitral stenosis complicated with small left ventricle are mostly in the range of normal or slight reduction; so, the changes before and after operation are not obvious; (2) although the baseline values of LVEF and LVFS are mostly in the normal range, the left ventricular systolic function is not significantly improved in the short-term after operation because of the long course of disease, preoperative myocardial involvement to varying degrees, significant decline of myocardial reserve function, intraoperative surgical trauma, and myocardial ischemia-reperfusion injury; and (3) the results were also related to the subjective factors affecting the results of cardiac color echocardiography and the different sensitivities and specificities of LVEF and LVFS. Half a year after operation, the left ventricular systolic function was also improved with the increase of left ventricular return blood volume and the recovery of left ventricular morphology.

The article "Prognostic Value of Creatine Phosphate and Inflammatory Markers for Mitral Valve Replacement: A Systematic Review and Meta-Analysis" was retracted in 2023. Reasons: signs of a paper mill; suspected computer-generated content; unreliable results or conclusions; concerns about the data.

In the surgical treatment of rheumatic heart disease, mitral valvuloplasty has better short-term and long-term outcomes than replacement [17]. These advantages have not been fully confirmed because of the lack of prospective randomized controlled studies. Due to the limitations of disease characteristics and ethics, it is difficult to implement prospective randomized controlled study in clinic. At present, the results of small sample noncontrolled studies are the main reference basis for optimizing the operation, which makes it necessary to summarize high-quality studies related to rheumatic heart disease and conduct systematic evaluation.

At present, the research of transcatheter mitral valve replacement still stays in the research of instruments and early clinical effects, and there is no powerful research that can really promote transcatheter mitral valve replacement to practical clinical application [18]. Although the current transcatheter mitral valve replacement can meet the basic requirements, such as adapting to complex anatomical positions, good valve function, improvement of perivalvular leakage, and gradual reduction of short-term complications, there are still many gaps and challenges in the long-term complications such as valve thrombosis, valve durability, and cardiac function damage [19]. Reviewing the process from doubt to popularization of transcatheter mitral valve replacement technology, we have reason to believe that with the development of bioengineering and catheter technology, better valve structure design and clinical results of transcatheter mitral valve replacement are bound to appear and finally serve the majority of patients.

Creatine phosphate is an important effector molecule in response to the activation of energy metabolism system [20]. This study found that the level of Ang II in the experimental group was significantly higher than that in the control group, which was consistent with the current foreign related studies. Creatine phosphate can promote the division and proliferation of fibroblasts and the synthesis of type 1 and 2 collagen. The process of cardiac atrial remodeling is similar to that of ventricular interstitial remodeling. The same process of cardiac fibroblast proliferation leads to collagen remodeling. Creatine phosphate may play an important role in the pathogenesis of atrial fibrillation through atrial fibrosis remodeling [21, 22].

The role of inflammation theory in the pathogenesis of atrial fibrillation is a research hotspot in recent years. CRP represents an important indicator of inflammatory response and has high sensitivity. It can indicate the degree of local or systemic tissue inflammation, which has been used in clinical practice. IL-6 is a multifunctional cytokine that regulates immune response and inflammatory response [23]. This study found that CRP and IL-6 in the experimental group of rheumatic heart disease with simple mitral stenosis and atrial fibrillation were significantly higher than those in the control group of rheumatic heart disease with simple mitral stenosis and sinus rhythm, which was consistent with previous studies [24]. Foreign studies have found that the level of CRP in vivo is related to the load of atrial fibrillation. With the step-by-step increase of CRP concentration, the load of atrial fibrillation is also gradually increasing. It is suggested that the inflammatory effects of CRP and IL-6 may play an important role in the pathogenesis of atrial fibrillation [25].

The article "Prognostic Value of Creatine Phosphate and Inflammatory Markers for Mitral Valve Replacement: A Systematic Review and Meta-Analysis" was retracted in 2023. Reasons: signs of a paper mill; suspected computer-generated content; unreliable results or conclusions; concerns about the data.

## 5. Conclusions

Correlation analysis showed that creatine phosphate, CRP, and IL-6 were positively correlated with left atrial diameter and negatively correlated with LVEF, further suggesting that creatine phosphate and inflammatory cytokines play an important role in the process of cardiac insufficiency. It is found that creatine phosphate can promote inflammatory response and increase the expression of proinflammatory cytokines. There is a synergistic effect between phosphocreatine and inflammatory response: phosphocreatine promotes inflammation, and inflammation itself can also activate phosphocreatine, thereby increasing the expression of Ang II. However, it should be noted that in order to explore the exact role of creatine phosphate and inflammatory response in the pathogenesis of valvular atrial fibrillation, further large-scale basic and clinical research is needed.

## Figures and Tables

**Figure 1:** ROC curves of RCTs.

**Figure 2:** Comparison of intraoperative cardiac beat rate between the phosphocreatine group.

**Figure 3:** Comparison of CK-MB levels in venous blood 24 h after aorta occlusion between the creatine phosphate group and control group.

**Figure 4:** Funnel plot of included studies demonstrating the odds ratios of 30-day mortality in the mitral valve repair group compared to mitral valve replacement group. SE: standard error.

**Table 1:** Basic characteristics of included literature.

Inflammatory marker		
Literature	Document	15% different from the heart rate
Soluble molecules, such as the content and selection of adhesive cells	Changed	The survey is 15%
Cytokines	Changed	Less than 100% contaminated and 15% in other conditions
HS-CRP	Stable	>15%
LVEVDI	Changed	100% explosives
RBC, HBC, and other values	Stir	18%
LVEVDI	Stable	80%
Proenzymes such as CK-MB and proatherogenic enzymes	Stir	100%
C-reactive protein	Changed	80%

The article "Prognostic Value of Creatine Phosphate and Inflammatory Markers for Mitral Valve Replacement: A Systematic Review and Meta-Analysis" was retracted in 2023. Reasons: signs of a paper mill; suspected computer-generated content; unreliable results or conclusions; concerns about the data.

**Table 2:** Statistics.

Study name	Propensity score matching	No. of participants (repair)	No. of participants (replacement)
DiGregorio (2004)	No	46	13
Ailawadi (2008)	No	70	47
Chikwe (2011)	Yes	227	95
Nloga (2011)	No	75	54
Silaschi (2016)	Yes	63	63
Chivasso (2017)	No	150	97
Farid (2019)	Yes	78	78
Seese (2020)	No	301	171

**Table 3:** Statistical data of prognostic factors.

Index	No response rate	95% CL	Sum *P*
Bilirubin (mg/dL)	1.054	1.026	0.0001
HGB (g/dL)	0.694	0.600-0.802	0.0001
HS-CRP (mg/dL)	2.654	1.546-4.506	0.0001
IL10	3.506	2.571-4.782	0.0001
IL6	0.403	0.260-0.624	0.0001
Creatine phosphate	1.450		

## Data Availability

The data underlying the results presented in the study are available within the manuscript.
